The article "Comparison of the effects of EGF, FGF-b, and NGF on the proliferation, migration, and reprogramming of primary rat Müller cells" was retracted in 2024. Reasons: unreliable data; concerns about the data.

# Comparison of the effects of EGF, FGF-b, and NGF on the proliferation, migration, and reprogramming of primary rat Müller cells

**DOI:** 10.3389/fncel.2024.1338129

**Published:** 2024-02-21

**Authors:** Yanying Liao, Miaoqin Wu

**Affiliations:** ^1^Hangzhou Medical College, Hangzhou, Zhejiang, China; ^2^Center for Rehabilitation Medicine, Department of Ophthalmology, Zhejiang Provincial People's Hospital (Affiliated People's Hospital), Hangzhou Medical College, Hangzhou, Zhejiang, China

**Keywords:** growth factors, Müller, proliferation, migration, reprogramming

## Abstract

**Purpose:**

During the healing process of full-thickness macular holes (FTMHs), the closure and recovery of the hole depend on the migration, proliferation, and activation of Müller cells to promote the closure of holes and restoration of the photosensitive layer. In this study, we investigated the ability of the epidermal growth factor (EGF), fibroblast growth factor-basic (FGF-b), and nerve growth factor (NGF) to influence this process by regulating proliferation, migration, and reprogramming of primary rat Müller cells.

**Methods:**

Cell proliferation was measured using CCK8 [2- (2-Methoxy-4-nitrophenyl)-3- (4-nitrophenyl)-5- (2,4-disulfophenyl)-2H-tetrazolium Sodium Salt] colorimetric assays and EdU [5-Ethynyl-2′-deoxyuridine] assays over 48 h. Cell migration was measured using scratch-wound assays and transwell migration assays over 48 h. In addition, we conducted Western blot assays and immunofluorescence assays on cells that were specially treated for 1, 3, and 5 days for cell reprogramming. The percentage of EdU-positive cells in Nestin-positive have also been tested by co-immunofluorescence (Co-IF) staining.

**Results:**

EGF and FGF-b significantly promoted the proliferation of Müller cells (*p* < 0.05) at a concentration of 0–50 ng/mL, but NGF did not (*p* > 0.05), compared to untreated controls. Exogenous FGF-b and EGF promote the reprogramming of primary rat Müller cells, significantly enhancing the neural stem cell marker Nestin after stimulation on the 1st, 3rd, and 5th days, respectively. The expression of Müller cell marker Vimentin was significantly (*p* < 0.05) reduced during this period compared to the control group. However, there was no significant difference between the NGF and control groups. Furthermore, the EGF group expressed stronger Nestin expression than the SCM group. The Co-IF staining showed that early 50% of activated cells came from newly proliferating cells on the 5th day.

**Conclusion:**

These observations suggest that FGF-b can promote the activation of Müller cells in a short time and enhance the possessive features of neural stem cells, while EGF may act for a longer period of time. This may further the understanding of growth factor therapy in treating FTMHs, and Müller glia may be promising candidates for cell replacement therapy.

## Introduction

Full-thickness macular hole (FTMH) is a defect in the central fovea of the retina that can lead to severe vision deterioration (Gross, 2005; Michalewska et al., 2010; Duker et al., 2013; Chatziralli et al., 2018). At present, the treatment methods for FTMHs are mostly surgeries (Duker et al., 2013), and the closure rate of the hole after standard treatment is 85–90% (Gross, 2005), but there are still some refractory FTMHs that are not closed or the improvement of visual function is poor (Michalewska et al., 2010).

Müller cells are a special type of glial cells that span the entire depth of the neuroretina (Goldman, 2014). In the mature retina, they are anatomically and functionally essential for retinal development and homeostasis, serving as supporting cells for the neurons of the retina. Müller cells also play an important role in the recovery process of FTMH. Studies have shown (Kitao et al., 2019) that Müller cell proliferation and migration promote closure of FTMH, and the reconstruction of External Limited Membrane (ELM) and Ellipsoid Zone (EZ) layers relies on Müller cell migration to the ELM and EZ and then redifferentiation into photoreceptor cells (PC) including cone and rod cells. Many studies have reported that Müller cells tend to reprogram, possessing stem cell characteristics and differentiating into retinal nerve cells when retinal damage is in lower vertebrates and amphibians (Qin et al., 2009; Nagashima et al., 2013). However, for mammals, Müller glial cells hardly reprogram to produce neurons unless stimulated by exogenous cytokines or growth factors (Goldman, 2014; Gao et al., 2021).

Müller cells tend to secrete a variety of neurotrophic factors and cytokines (Wan et al., 2014), especially when injured, and these cells can be coaxed to proliferate and generate neurons under these special circumstances. Therefore, in this study, we used *in vitro* primary rat Müller cell models to further study the potential for epidermal growth factor (EGF), fibroblast growth factors-basic (FGF-b), and nerve growth factor (NGF) to regulate cell dose-related proliferation, migration, and reprogramming which might provide helpful hints to improve therapy for FTMHs in the long run. Few researchers have compared them together and explored their effects on cell proliferation, migration, and reprogramming, although previous studies have investigated the effects and mechanisms of one growth factor on Müller cells.

In this article, experiments were divided into four sections: (1) In the first part of this article, we used immunofluorescence (IF) to identify the purity of Müller cells. Vimentin, glutamine synthetase (GS), and CRALBP are specific proteins of Müller cells (Zalis et al., 2017); (2) In the second part, we tried to measure and compare the dose–response of EGF, FGF-b, and NGF on cell proliferation for Müller cells; (3) In the third part, we compared the effects of EGF, FGF-b, and NGF at a concentration of 10 ng/mL for migration of Müller cells. Few researchers have studied the migration of Müller cells, but it may be vital for the healing of FTMHs; (4) In the fourth part, we tested the effects of the EGF, FGF-b, NGF, and stem cell medium (SCM) groups on Müller cell reprogramming. As a specific marker of neural stem cells, the Nestin protein will be further studied for its expression changes. (5) In the last part of the study, based on previous results, we co-stained Müller cells under the effects of various growth factors with different markers and analyzed the proportion of proliferating cells in reprogrammed cells.

## Materials and methods

### Materials

Primary Müller cells from rat retina were obtained from CHI SCIENTIFIC, China; DMEM/F12 complete medium containing HEPES, 2 mM Alanyl-glutamine, 100 U/mL penicillin, 100 μg/mL streptomycin, and 10% FBS were obtained from Pricella, China; 100 × N_2_ supplement was obtained from GIBCO; recombinant human beta-NGF, FGF-b, and EGF were obtained from Novoprotein, China; primary antibodies against Glutamine Synthetase (GS), Vimentin, CRALBP, and Nestin were obtained from Abcam, USA; secondary antibodies was obtained from Proteintech, China; The Cell Counting Kit 8 (CCK8), Trypsin–EDTA (0.25%), Normal Goat Serum, and 5. 5-Ethynyl-2′-deoxyuridine (EdU) proliferation kit were obtained from Yeasen, China; 10 × PBS was obtained from Absin, China; Poly-D-lysine, 10% Triton X-100 Solution, 4% Paraformaldehyde Fix Solution, and antifade mounting medium with 4,6-diamidino2-phenylindole (DAPI) were obtained from Beyotime, China.

### Cell treatment

Müller cells of the P0 generation were dissociated using Trypsin–EDTA (0.25%) and cultured in DMEM/F12 complete medium [supplemented with 10% heat-inactivated fetal bovine serum (FBS) and maintained in a humidified incubator at 37°C with 5% CO_2_]. P2-P3 cells will be used for subsequent experiments. Primary Müller cells grown to confluence were then cultured in a serum-free medium (SFM; 50 units/mL penicillin, 50 units/mL streptomycin, 2 mmol-glutamine, and DMEM/F12 medium) for 12 h. The cultured cells were exposed to relevant concentrations of EGF, FGF-b, and NGF. For dedifferentiation, Müller cells were exposed to EGF, FGF-b, and NGF at concentrations of 10 ng/mL and stem cell medium (SCM, 20 ng/mL EGF, 10 ng/mL FGF-b) for 1, 3, and 5 days after starvation by SFM. 1 × N2 supplement was added to all groups.

### Identification of Müller cells

The IF method was used to identify primary rat Müller cells. Cells were cultured on glass coverslips and incubated with 10 ug/ml poly-L-lysine. Then, the cells were fixed in chilled 4% paraformaldehyde in 0.1 M PBS (pH 7.4) for 15 min and washed 3 times with PBS. The cells were permeabilized with 0.1% Triton X-100 in PBS for 15 min. Fixed cells were preincubated for 30 min in PBS containing 10% normal goat serum at room temperature, followed by incubation with various primary antibodies at 4°C overnight and detected using fluorescein-conjugated secondary antibody anti-rat or rabbit IgG (1:250) at room temperature for 2 h in the dark. The cells were stained with an antifade mounting medium with DAPI to visualize the nuclei. Eight visual fields were selected for positive statistics for each type of fluorescence staining (100× or 200×). The total number of nuclei counted in each marker was 303 (CRALBP), 484 (GS), and 758 (Vimentin). The manual counting method was used to calculate the number of positive cells (N_1_) and the total number (N_2_) of cells. The positive rate was % = N_1_/N_2_ × 100%.

### CCK8 assays

We measured the dose–response of EGF, FGF-b, and NGF on cell proliferation for Müller cells. Müller cells were seeded at a concentration of 4 × 10^4^ cells/ml in 96-well plates and grown for 24 h in DMEM/F12 medium. Cells were treated with EGF, FGF-b, and NGF at concentrations of 0, 0.5, 1, 5, 10, 20, 30, 40, and 50 ng/mL (*N* = 3 wells/concentration). The experiment was repeated three times (*N* = 9 wells total). After 48 h, 100 μL of the mixture (cck8 reagent: DMEM/F12 medium = 1:10) was added to each well and then incubated at 37°C for 1 h in the dark. Absorbance was measured at a wavelength of 450 nm. The 0 ng/mL treatment group is the control group, and the average absorbance of each experiment is A_avg_. The treated group was normalized by C_avg_, and dose–response curves were then plotted for each treatment.

### EdU assays

Müller cells were planted in 6-well plates, with 1 × 10^5^ cells per well. Growth factors were added to each group to achieve a final concentration of 10 ng/mL. After 24 h, the EdU working solution was added to each group, and the final concentration was 10 μM. Cells were fixed with 4% paraformaldehyde for 15 min, and the membrane was broken with 0.1% Triton-100 (diluted by PBS) for 15 min. A click reactive solution was prepared according to the instructions and added to the cells. After incubating in the dark for 30 min at room temperature, we observed and took photos under an inverted fluorescence microscope. Each group adopted six visual fields, and the fluorescence intensity of EdU was calculated (treated group: *F*_t_, control group: *F*_c_) using ImageJ software. Relative fluorescence intensity expression was *F*_t_/*F*_c_.

### Scratch-wound assays

Cells were seeded in six-well plates at a concentration of 1 × 10^5^ cells/ml and grown for 3 days to approximately 85% confluence in DMEM/F12 medium, followed by a 12-h adaptation in SFM. Wounds were then made in confluent cell monolayers using a 1-ml pipette tip and drawn vertically across the center of the well. All wounds were made by an independent researcher (YL). Wells were then gently washed three times with PBS to remove any cell debris and treated with EGF, FGF-b, NGF, or PBS. The concentration of each growth factor is 10 ng/ml. Wound areas were observed at *T* = 0, 24, and 48 h post scratch, and then images of wound areas were captured using a 5 × objective. Three images were collected for each hole. Every experiment was repeated three times on separate occasions, giving a total of *N* = 9 images for analysis for each condition. The treated group migration area (S_t_) was normalized by control group migration (S_c_). The order of growth factors administration and wounding within the 6-well plates were randomized for each experiment to minimize bias.

### Transwell migration assays

In SFM, 100 μL Müller cell suspension (1 × 10^4^ cells) is placed on the upper layer of a cell culture insert with a permeable membrane, and a DMEM/F12 medium containing 10% FBS and EGF or FGF-b or NGF or PBS (control group) is placed below the cell permeable membrane. Following a 48-h incubation period, the cells that migrated through the membrane were stained by 0.1% purple crystal dye solution and counted. Relative migration was the number of cell migrations in the treated group (*N*_t_)/the number of cell migrations in the control group (*N*_c_).

### IF staining assays

The operation process is consistent with Müller cell identification, and the fluorescence intensity of images was analyzed using ImageJ software. Relative fluorescence intensity was the fluorescence intensity of the treated group (*F*_t_)/fluorescence intensity of the control group (*F*_c_).

### Western blot assays

Cells were lysed by RAPI lysis buffer on ice to extract total cell protein. SDS-PAGE separated 25 μg of total protein lysates, and specific primary antibodies detected the expression levels of different proteins. After being hatched with HRP-conjugated secondary antibody for 1 h, we captured ECL images using an X-ray film. The grayscale of targeted bands was normalized to the grayscale of Vinculin or GAPDH.

### Co-IF staining assays

Cells were treated with EGF and FGF-b after starvation, and 10 μM of EdU was added at 0, 48, and 96 h, respectively. IF staining and click reactive solution were performed simultaneously after 24 h **of each** time point. The percentage of positive cells was the percentage of EdU+ cells in Nestin+ cells, which was counted using ImageJ software. Nine visual fields were selected for statistics and repeated three times.

### Statistical analysis

All experiments were performed at least in triplicate, with results shown as means ± standard deviation. All images were analyzed using ImageJ software and GraphPad Prism 9.4.0. All vector maps were drawn using GraphPad software. A one-way ANOVA test was used to evaluate statistical significance. For all tests, a *p*-value less than 0.05 was considered to be statistically significant. All *p*-values given were the results of two-sided tests.

## Results

### Identification of Müller cells

The IF staining showed that the proportion of specific proteins expressed in primary rat Müller cells was over 95% (CRALBP: 95.76%, GS: 99.60%, Vimentin: 96.00%, respectively) (Figure 1).

**Figure 1:** Purity identification of Müller cells: immunocytochemical analysis showed that >95% **(J)** of purified cells expressed immunoreactivities corresponding to Müller cell markers (**A–F**, Scale bars, 125 μm; **G–I**, Scale bars, 275 μm.), **(A–C)** CRALBP, **(D–F)** GS, and **(G–I)** Vimentin.

### Effects of growth factors on the proliferation of Müller cells

To test the ability of EGF, FGF-b, and NGF to promote cell proliferation, we carried out the experimental design shown in Figure 2A. Primary Müller cells in P3-P4 were cultured for 24 h, and then EdU was added to distinguish their progeny from the surviving post-mitotic cells. After adding the click reactive solution, it showed that the EGF and FGF-b groups have more mitotic neonatal cells (Figures 2B–M). Quantification of relative EdU fluorescence expression for each treatment showed that the EGF and FGF-b groups had a significantly (*p* = 0.0035, *p* < 0.0001, respectively, Figure 2N) higher ability of proliferation than the control group. However, the NGF group had minimal proliferation with no significant effect (*p* > 0.9999). For CCK8 assays, FGF-b-treated and EGF-treated Müller cells showed a dose-related (0–50 ng/mL) increase, and the FGF-b group showed a stronger proliferative capacity than the EGF group (Figure 2O). However, for all concentrations of NGF (0–50 ng/mL), Müller cell proliferation did not differ from untreated cells at 48 h (Figures 2A,B).

**Figure 2:** The ability of EGF, FGF-b, and NGF to promote cell proliferation. **(A–M)** Cell proliferation was detected by EdU under the NGF, EGF, and FGF-b at a concentration of 10 ng/mL. **(A)** Experimental design. **(B–D)** Control group, **(E–G)** NGF group, **(H–J)** EGF group, **(K–M)** FGF-b group (Scale bars, 125 μm, *n* = 3). **(N)** Quantification of relative EdU fluorescence expression for each treatment (*n* = 10), **p < 0.01, ****p < 0.0001. **(O)** The relationship between the concentration (0, 0.5, 1, 5, 10, 20, 30, 40, and 50 ng/mL) of each growth factor and proliferation at 48 h (*n* = 3).

### Effects of growth factors on the migration of Müller cell

Cell migration *in vitro* was measured using transwell and scratch-wound assays, with various patterns of wound healing observed for each growth factor (Figure 3). Transwell assays showed that FGF-b-treated and EGF-treated cell migration numbers were significantly higher than untreated cells at 48 h (*p* < 0.0001, Figures 3A–D,M). Quantification of EGF**-** and FGF-b**-**treated Müller cells displayed rapid migration (Figures 3E–L,N,O) into the wound area at both 24 h (*p* = 0.0064 < 0.01 and *p* < 0.0001, respectively) and 48 h (*p* = 0.0025 < 0.01 and *p* < 0.0001, respectively), and individual cells were observed in the central of the wound area. However, for the NGF and untreated group**s**, most cell bodies remain at the edge of the wound (Figures 3E–L). The number of migration and relative migration area of cells in the NGF group were similar (*p* > 0.05, Figure 3) to those in the untreated group, both in transwell and scratch-wound assays.

**Figure 3:** Comparison of migration number or area in EGF, FGF-b, and NGF treated and control groups for Müller cells. **(A–D)** The cells that migrated through the membrane, *T* = 48 h. **(M)** Number of migrations of Müller cells at 48 h. Scale bars, 125 μm. **(E–L)** Wound areas at *T* = 24 and 48 h (red sections) compared to areas at *T* = 0 (yellow dashed line) for Müller cells. Scale bars, 200 μm. **(M)** Quantification of Transwell assays (*T* = 48 h, *n* = 3). **(N,O)** Quantification of Scartch-wound assays (**N**: *T* = 24 h, **O**: *T* = 48 h; both *n* = 3). The concentration of growth factor: 10 ng/mL. **p < 0.01, ****p < 0.0001.

### Effects of growth factors on the reprogramming of Müller cells

A large proportion of the EGF-treated and FGF-b-treated cells showed a distinct neural morphology, with longer neurites and small phase bright cell soma characteristic of neurons which is similar to the SCM group. However, the control and NGF groups didn’t show the characteristic of neurons (Figures 4A–D). Depending on the different growth factors used for differentiating cells cultured in SFM, there was also variability in the fluorescence expression markers of neural stem cells and Müller cells (Figures 4F–T). Staining for Nestin, a progenitor and neural stem cell marker, was observed in cells cultured with EGF, FGF-b, and SCM, but very little or no staining was observed in cells cultured in the absence of these factors (Figures 4F–J). Quantification of IF showed the FGF-b group had a higher expression of Nestin (*p* < 0.0001) and lower expression of Vimentin protein (*p* = 0.0034 < 0.01) than the untreated group and even the SCM group after 1 day of drug stimulation. Meanwhile, the EGF group expressed lower Vimentin protein (*p* = 0.0089 < 0.01) but a similar Nestin protein (*p* > 0.05) than the untreated group on the 1st day. However, there was no significant difference in Nestin protein expression or Vimentin protein expression (both *p* > 0.05) between the NGF and the control groups (Figures 4U,V). Furthermore, the EGF group showed a higher expression of Nestin than the control (*p* = 0.0024 < 0.01, *p* = 0.001 < 0.01, respectively) on the third and fifth days. Three days after administration, the expression level of Nestin protein in the EGF group was even higher than that in the SCM group (*p* = 0.0039 < 0.01). The FGF-b (*p* = 0.0036 < 0.01, *p* < 0.0001, respectively) and SCM groups (*p* = 0.0029 < 0.01, *p* < 0.0001, respectively) showed significantly lower expression of Vimentin than the control group on the third and fifth days (Figures 4X,Z). The EGF group also showed lower (*p* < 0.0001) Vimentin expression on the fifth day. Western blots of Müller cell lysates showed that the expression of Nestin in the FGF-b and SCM groups was significantly increased (*p* = 0.0007 < 0.001, *p* = 0.0015 < 0.01, respectively) (Figures 5A,B) after the first day of growth factor cultivation. Nevertheless, the expression of Nestin in the EGF group was significantly increased (*p* = 0.0048 < 0.01) after 3 days of administration. The EGF group also expressed higher than the control group on the fifth day (*p* = 0.0015 < 0.01) as well as that in cells cultured in SCM (*p* = 0.0379 < 0.05) (Figures 5A,D). For the NGF group, there was no significant increase (*p* > 0.05) in Nestin protein expression compared to the untreated group on the first, third, or fifth day of administration. Correspondingly, the EGF (*p* = 0.0032 < 0.01), FGF-b (*p* = 0.0272 < 0.05), and SCM groups (*p* = 0.0262 < 0.05) showed lower expression of Vimentin protein than the control group, while the NGF group did not (*p* > 0.05) (Figures 5E,F).

**Figure 4:** Dedifferentiation of Müller cells and fluorescence expression of its specific biomarkers. **(A–E)** Phase contrast micrographs of Müller cells on 1 day after different treatments. Scale bars, 200 μm. **(F–J)** Fluorescence expression of stem cell biomarker (Nestin) in cells (*n* = 3). **(K–O)** Fluorescence expression of Müller cells biomarker (Vimentin) in cells (*n* = 3). **(P–T)** Merged. Scale bars, 125 μm. **(U–Z)** Quantification of immunofluorescence showing expression of Nestin and Vimentin proteins (**U,W,Y**: Nestin; **V,X,Z**: Vimentin) *p < 0.05, **p < 0.01, ***p < 0.001,****p < 0.0001.

**Figure 5:** Dedifferentiation of Müller cells and Western blot showing its specific biomarkers. **(A)** Representative Western blot of Müller cells showing the expression of neural stem cell biomarkers (Nestin protein) in each group. **(B–D)** Quantification of Western blots showing expression of Nestin protein (both *n* = 3). **(E)** Representative Western blot showing the expression of Müller cell biomarkers (Vimentin protein) in each group. **(F)** Quantification of Western blots showing expression of Vimentin protein (*n* = 3). *p < 0.05, **p < 0.01, ***p < 0.001.

### Relationship between proliferation and activation of Müller cells

To test the percentage of proliferating cells in active Müller cells, we carried out the experimental design detailed in Figure 6A. Co-IF staining showed 32.44 ± 6.40%, and 46.65 ± 7.72% of reprogramming cells presented EdU+ (EdU+/Nestin+) after 1 day of EGF and FGF-b stimulation (Figures 4B–J), respectively. On the 3rd day, we observed 16.36 ± 1.99% (EGF) and 12.92 ± 1.50% (FGF-b) of cells expressed EdU+/Nestin+ (Figure 4K). In addition, 47.26 ± 7.17% (EGF) and 45.79 ± 2.90% (FGF-b) of cells expressed EdU+/Nestin+ after 5 days of stimulation (Figure 4L).

**Figure 6:** Co-IF staining of EdU (red), Nestin (orange), Gail cell markers (green), and DAPI (blue). BrdU-tagged cells from active Müller cells (EdU+/Nestin+, white arrows). **(A)** Experimental design. **(B–I)** Co-IF staining of EdU, Nestin, and Vimentin after 1 day of EGF and FGF-b stimulation. **(J–L)** The percentage of EdU+ cells in Nestin+ cells on 1, 3, and 5 days, respectively (*n* = 3, nine visual fields were selected for each repetition for statistics).

## Discussion

FTMH is a vital cause of central visual loss worldwide, with an estimated incidence of 7.8 persons/100,000 population per year (Wang et al., 2006). Müller cells are the primary macro-glial cells, accounting for 90% of the human retinal glial cells (Goldman, 2014; Chen et al., 2018). They play a major role in maintaining the integrity of the retina and the normal functioning of the metabolic environment, including retinal wound healing, such as FTMHs (Kitao et al., 2019). The ability of cells to proliferate, migrate, and reprogram is part of the FTMH-healing process (Wakabayashi et al., 2010; Kitao et al., 2019), so growth factors that encourage the replication and activation of Müller cells should be considered.

It has been proven that there are multiple receptors for growth factors in the eye, such as EGF, FGFs, NGF, insulin, insulin-like growth factors (IGFs), and transforming growth factor-β (TGF-β) (Goldman, 2014). Cell cycle reentry can often be stimulated and maintained via exposure to extracellular factors such as EGF, FGF-b, IGF, and TGF-β, which have been proven to be vital in characterizing progenitor potential. As a potent mitogen for Müller cells, the previous study confirmed that EGF stimulates Müller cell proliferation via a BMP-dependent mechanism (Ueki and Reh, 2013). Nickerson et al. (Nickerson et al., 2011) demonstrate that cotreatment with EGF and EPO suppresses aspects of EGF-induced glial reactivity, alters the retinal distribution of BrdU-positive nuclei, and might regulate the expression of developmental phenotypes seen in these cells. FGF-b, expressed by photoreceptors, other retinal cells, and the central nervous system, enhances endothelial cell proliferation, migration, and survival (Gao and Hollyfield, 1995). Studies (Romo et al., 2011) have shown that FGF-b may promote the establishment and maintenance of avascular zones in primates.

Lawrence et al. (2007) revealed that Müller cells can form neuro-spheres and express neural stem cell markers in the presence of extracellular matrix and FGF-b. Nerve growth factors (NGFs) are well-known as a classic neuroprotective factor that has a protective effect on Müller cells to relieve retinal gliosis in rats via the Trk-A signaling pathway (Sun et al., 2008). Liu et al. reported that NGFs, produced by Müller cells, also play a critical role in retinal neovascularization (Liu et al., 2010).

In the present study, we focused on the proliferative and migratory potentials and the ability to reprogram and obtain stem cell characteristics of primary rat Müller cells in various environments (EGF, FGF-b, and NGF treated). We found that EGF and FGF-b might significantly promote the proliferation and migration of Müller cells and also activate Müller cells, which promoting their reprogramming into pluripotent stem cells.

The ability of cells to proliferate is the first part of the wound-healing process, as shown in Figure 1. We discovered that EGF and FGF-b significantly promote the proliferation of Müller cells (Figure 3, *p* < 0.05), but NGF does not (*p* > 0.05). For the FGF-b group, the effect of enhancing the Müller cell proliferation at concentrations of 0–50 ng/mL is greater than the EGF culturing group (Figure 3O). Previous studies confirmed that growth factors may stimulate Müller glial cell proliferation acting through Notch as well as FGF receptor, EGF receptor, mitogen-activated protein kinase (MAPK), and extracellular signal-regulated kinase (ERK) signaling pathways (Fischer et al., 2002, 2009; Ghai et al., 2010). In addition, the current study (Oh et al., 2013) suggests that appropriate gliosis can promote FTMH healing, but excessive gliosis may affect the bridging of the ELM and EZ, which might greatly impair visual function. Although the potential molecular mechanisms need further clarification, our data may indicate that growth factors have different abilities to promote cell proliferation and might provide further insights into the closure of FTMH by growth factors.

In addition to proliferation, migration is a vitally important part of the initial process of FTMH wound healing (Figure 1; Wu et al., 2021). Our data revealed that EGF and FGF-b increased the migration of Müller cells at a concentration of 10 ng/mL (Figure 5), both for vertical (transwell assays) and horizontal migrations (scratch-wound assays). Bringmann et al. proposed that activation of p38 MAPKs (Bringmann et al., 2009) is a possible mechanism to direct Müller cell migration, and the migratory effects of FGF-b are mediated through direct activation of p38 MAPKs, while EGF stimulates the EGF receptor tyrosine kinase that eventually activates p38 MAPKs. Recent findings also imply that Sox11b plays key roles in MGPC migration and fate determination during retina regeneration in zebrafish (Song et al., 2023). Furthermore, studies confirmed that bFGF and insulin lead to the migration of Müller glia to the photoreceptor layer (Goel and Dhingra, 2021). Based on these observations, we have confirmed that these selected factors aid the migration ability of Müller cells and might promote the rearrangement of ELM and EZ layers, providing the possibility of improving visual function.

In addition, stimulating Müller glia causes them to undergo a reprogramming event and acquire stem cell characteristics that enable them to generate progenitors for retinal repair, providing greater possibilities for improving visual function (Figure 1; Lawrence et al., 2007). We have demonstrated that the FGF-b and SCM groups showed strong stem cell characteristics, 1 day after administration (Figures 6, 7). The EGF and SCM groups showed high expression of the stem cell biomarker (Nestin) 3 and 5 days after administration (Figures 7A–D); however, the FGF-b cultured cells lost stem cell characteristics. Correspondingly, the features of mature Müller glia were reduced, and the expression of the Vimentin protein decreased (Figures 7E,F). These observations indicate that FGF-b can promote the activation of Müller cells in a short time and enhance the possessive features of neural stem cells, and EGF might act for a longer time. As we can see, SCM did not show any advantages over EGF and FGF-b treatments (Figures 6, 7). Furthermore, we found that nearly 50% (EGF: 47.26 ± 7.17%, FGF-b: 45.79 ± 2.90%) of Nestin+ cells were simultaneously positive for EdU expression on the 5th day (Figure 4L), indicating that nearly 50% of activated cells came from newly proliferating cells.

**Figure 7:** Mechanism illustration of growth factors used for macular hole repair.

As for differentiation, previous studies showed that Mps1, the galectin Drgal1-L2 (Craig et al., 2010), FGF signaling (Qin et al., 2011), Notch signaling (Wan et al., 2012), *N*-cadherin (Nagashima et al., 2013), and Insm1a (Ramachandran et al., 2012) seem to promote the differentiation of Müller cells in zebrafish. Even if mammalian Müller glia could be reprogrammed, the progenitor formation and differentiation into neurocytes is always prevented (Goldman, 2014). Lawrence et al. (Lawrence et al., 2007) and Das et al. (Das et al., 2006) attempted to cultivate mammalian Müller cells using FGF2, retinoic acid (RA), and brain-derived neurotrophic factor (BDNF), which seemed to promote the regeneration of ganglia, bipolar cells, and photoreceptors. Some studies (Araki et al., 2007) suggest that EGF can enhance the possibility of pineal cells differentiating into photoreceptor cells. However, the mechanisms that control the differentiation of mammalian Müller cell-derived progenitors in adult retina are still poorly understood.

Zhang et al. (2019a,b) revealed that human Müller cells co-cultured with ILM or NGF promoted cell proliferation and transdifferentiation via the PI3K/Akt pathway. However, we found that NGF did not promote the proliferation (Figure 2) and activation (Figures 4, 5) of primary rat Muller cells, and this difference may be caused by differences in cell types. As a neuroprotective factor, NGF may play an important role in the maintenance and support of other retinal cell types in the retina (Telegina et al., 2019).

Astrocytes, which also provide a structural scaffold (Reichenbach and Bringmann, 2020) for the fovea, mediate traction changes in the fovea and have a positive effect on protecting the fovea and its regeneration, as well as the Müller cells. Retinal damage caused by FTMH can lead to glial hyperplasia, involving the hypertrophy, proliferation, and migration of Müller cells and astrocytes, which may lead to the formation of glial scars (Bringmann et al., 2009). The formation of temporary glial cells is a part of the regeneration of the central fovea after FTMH surgery closure (Oh et al., 2010), while persistent glial scars (Oh et al., 2010; Kitao et al., 2019) hinder the regeneration of the central fovea.

The current research has several limitations. One is that we only studied three common growth factors, and other growth factors, such as IGFs, BDNF, and TGF-β, were not included in the study. Second, there is still a lack of research on some regulatory mechanisms in this study. The last limitation is that despite being an *in vitro* study, we are aware that our study could not exclude the possibility of proliferative lesions *in vivo*. Therefore, further basic research *in vivo* was required to confirm whether reprogrammed Müller cells can differentiate into photoreceptors.

## Conclusion

Taken together, our results have further demonstrated that dose-dependent EGF and FGF-b can promote the proliferation and migration of Müller cells, which enables the manufacture of a microenvironment that supports wound healing in FTMHs. Moreover, Müller cell reprogramming (activated) and exhibiting neural stem cell characteristics have been shown to occur in EGF and FGF-b environments. This study adds to the growing recognition of the importance of generating Müller glial cell-derived progenitors under the stimulation of exogenous growth factors. Understanding the responsiveness of Müller glia to exogenous growth factors will be necessary for the development of effective cell replacement therapy and growth factors therapy.

## Data availability statement

The original contributions presented in the study are included in the article/supplementary material, further inquiries can be directed to the corresponding author.

## Ethics statement

Ethical approval was not required for the studies on animals in accordance with the local legislation and institutional requirements because only commercially available established cell lines were used.

## Author contributions

YL: Conceptualization, Data curation, Formal analysis, Investigation, Methodology, Software, Supervision, Visualization, Writing – original draft, Writing – review & editing. MW: Conceptualization, Funding acquisition, Investigation, Project administration, Resources, Validation, Visualization, Writing – review & editing.

## References

[ref1] ArakiM.SuzukiH.LayerP. (2007). Differential enhancement of neural and photoreceptor cell differentiation of cultured pineal cells by FGF-1, IGF-1, and EGF. Dev. Neurobiol. 67, 1641–1654. doi: 10.1002/dneu.20534, PMID: 17577207

[ref2] BringmannA.IandievI.PannickeT.WurmA.HollbornM.WiedemannP.. (2009). Cellular signaling and factors involved in Müller cell gliosis: neuroprotective and detrimental effects. Prog. Retin. Eye Res. 28, 423–451. doi: 10.1016/j.preteyeres.2009.07.001, PMID: 19660572

[ref3] ChatziralliI. P.TheodossiadisP. G.SteelD. H. W. (2018). Internal limiting membrane peeling in macular hole surgery; why, when, and how? Retina 38, 870–882. doi: 10.1097/IAE.000000000000195929210940

[ref4] ChenL.WeiY.ZhouX.ZhangZ.ChiW.GongL.. (2018). Morphologic, biomechanical, and compositional features of the internal limiting membrane in pathologic myopic foveoschisis. Invest. Ophthalmol. Vis. Sci. 59, 5569–5578. doi: 10.1167/iovs.18-24676, PMID: 30480705

[ref5] CraigS. E.ThummelR.AhmedH.VastaG. R.HydeD. R.HitchcockP. F.. (2010). The zebrafish galectin Drgal1-l2 is expressed by proliferating Müller glia and photoreceptor progenitors and regulates the regeneration of rod photoreceptors. Invest. Ophthalmol. Vis. Sci. 51, 3244–3252.20071673 10.1167/iovs.09-4879PMC2891476

[ref6] DasA. V.MallyaK. B.ZhaoX.AhmadF.BhattacharyaS.ThoresonW. B.. (2006). Neural stem cell properties of Müller glia in the mammalian retina: regulation by notch and Wnt signaling. Dev. Biol. 299, 283–302. doi: 10.1016/j.ydbio.2006.07.029, PMID: 16949068

[ref7] DukerJ. S.KaiserP. K.BinderS.de SmetM. D.GaudricA.ReichelE.. (2013). The international vitreomacular traction study group classification of vitreomacular adhesion, traction, and macular hole. Ophthalmology 120, 2611–2619. doi: 10.1016/j.ophtha.2013.07.042, PMID: 24053995

[ref8] FischerA. J.McGuireC. R.DierksB. D.RehT. A. (2002). Insulin and fibroblast growth factor 2 activate a neurogenic program in Müller glia of the chicken retina. J. Neurosci. 22, 9387–9398. doi: 10.1523/JNEUROSCI.22-21-09387.2002, PMID: 12417664 PMC6758014

[ref9] FischerA. J.ScottM. A.TutenW. (2009). Mitogen-activated protein kinase-signaling stimulates Müller glia to proliferate in acutely damaged chicken retina. Glia 57, 166–181. doi: 10.1002/glia.20743, PMID: 18709648 PMC2774719

[ref10] GaoH.HollyfieldJ. G. (1995). Basic fibroblast growth factor in retinal development: differential levels of bFGF expression and content in normal and retinal degeneration (rd) mutant mice. Dev. Biol. 169, 168–184. doi: 10.1006/dbio.1995.1135, PMID: 7750636

[ref11] GaoH. A. L.HuangX.ChenX.XuH. (2021). Muller glia-mediated retinal regeneration. Mol. Neurobiol. 58, 2342–2361. doi: 10.1007/s12035-020-02274-w, PMID: 33417229

[ref12] GhaiK.ZelinkaC.FischerA. J. (2010). Notch signaling influences neuroprotective and proliferative properties of mature Müller glia. J. Neurosci. 30, 3101–3112. doi: 10.1523/JNEUROSCI.4919-09.2010, PMID: 20181607 PMC2834965

[ref13] GoelM.DhingraN. K. (2021). bFGF and insulin lead to migration of Müller glia to photoreceptor layer in rd1 mouse retina. Neurosci. Lett. 755:135936. doi: 10.1016/j.neulet.2021.135936, PMID: 33910061

[ref14] GoldmanD. (2014). Muller glial cell reprogramming and retina regeneration. Nat. Rev. Neurosci. 15, 431–442. doi: 10.1038/nrn3723, PMID: 24894585 PMC4249724

[ref15] GrossJ. G. (2005). Late reopening and spontaneous closure of previously repaired macular holes. Am. J. Ophthalmol. 140, 556–558. doi: 10.1016/j.ajo.2005.03.04416139019

[ref16] KitaoM.WakabayashiT.NishidaK.SakaguchiH.NishidaK. (2019). Long-term reconstruction of foveal microstructure and visual acuity after idiopathic macular hole repair: three-year follow-up study. Br. J. Ophthalmol. 103, 238–244. doi: 10.1136/bjophthalmol-2017-311689, PMID: 29632001

[ref17] LawrenceJ. M.SinghalS.BhatiaB.KeeganD. J.RehT. A.LuthertP. J.. (2007). MIO-M1 cells and similar muller glial cell lines derived from adult human retina exhibit neural stem cell characteristics. Stem Cells 25, 2033–2043. doi: 10.1634/stemcells.2006-0724, PMID: 17525239

[ref18] LiuX.WangD.LiuY.LuoY.MaW.XiaoW.. (2010). Neuronal-driven angiogenesis: role of NGF in retinal neovascularization in an oxygen-induced retinopathy model. Invest. Ophthalmol. Vis. Sci. 51, 3749–3757. doi: 10.1167/iovs.09-422620207957

[ref19] MichalewskaZ.MichalewskiJ.AdelmanR. A.NawrockiJ. (2010). Inverted internal limiting membrane flap technique for large macular holes. Ophthalmology 117, 2018–2025. doi: 10.1016/j.ophtha.2010.02.01120541263

[ref20] NagashimaM.BarthelL. K.RaymondP. A. (2013). A self-renewing division of zebrafish Müller glial cells generates neuronal progenitors that require N-cadherin to regenerate retinal neurons. Development 140, 4510–4521. doi: 10.1242/dev.090738, PMID: 24154521 PMC3817940

[ref21] NickersonP. E.McLeodM. C.MyersT.ClarkeD. B. (2011). Effects of epidermal growth factor and erythropoietin on Müller glial activation and phenotypic plasticity in the adult mammalian retina. J. Neurosci. Res. 89, 1018–1030. doi: 10.1002/jnr.22629, PMID: 21484851

[ref22] OhJ.SmiddyW. E.FlynnH. W.GregoriG.LujanB. (2010). Photoreceptor inner/outer segment defect imaging by spectral domain OCT and visual prognosis after macular hole surgery. Invest. Ophthalmol. Vis. Sci. 51, 1651–1658. doi: 10.1167/iovs.09-442019850825

[ref23] OhJ.YangS. M.ChoiY. M.KimS. W.HuhK. (2013). Glial proliferation after vitrectomy for a macular hole: a spectral domain optical coherence tomography study. Graefes Arch. Clin. Exp. Ophthalmol. 251, 477–484. doi: 10.1007/s00417-012-2058-9, PMID: 22623115

[ref24] QinZ.BarthelL. K.RaymondP. A. (2009). Genetic evidence for shared mechanisms of epimorphic regeneration in zebrafish. Proc. Natl. Acad. Sci. U. S. A. 106, 9310–9315. doi: 10.1073/pnas.0811186106, PMID: 19474300 PMC2695073

[ref25] QinZ.KiddA. R.ThomasJ. L.PossK. D.HydeD. R.RaymondP. A.. (2011). FGF signaling regulates rod photoreceptor cell maintenance and regeneration in zebrafish. Exp. Eye Res. 93, 726–734. doi: 10.1016/j.exer.2011.09.003, PMID: 21945172 PMC3243491

[ref26] RamachandranR.ZhaoX. F.GoldmanD. (2012). Insm1a-mediated gene repression is essential for the formation and differentiation of Müller glia-derived progenitors in the injured retina. Nat. Cell Biol. 14, 1013–1023. doi: 10.1038/ncb2586, PMID: 23000964 PMC3463712

[ref27] ReichenbachA.BringmannA. (2020). Glia of the human retina. Glia 68, 768–796. doi: 10.1002/glia.2372731793693

[ref28] RomoP.MadiganM. C.ProvisJ. M.CullenK. M. (2011). Differential effects of TGF-beta and FGF-2 on in vitro proliferation and migration of primate retinal endothelial and muller cells. Acta Ophthalmol. 89, e263–e268. doi: 10.1111/j.1755-3768.2010.01968.x, PMID: 20670342

[ref29] SongK.LinZ.CaoL.LuB.ChenY.ZhangS.. (2023). Sox11b regulates the migration and fate determination of Müller glia-derived progenitors during retina regeneration in zebrafish. Neural Regen. Res. 18, 445–450. doi: 10.4103/1673-5374.346550, PMID: 35900444 PMC9396499

[ref30] SunX.XuX.WangF.ZhangX.HoP. C.LiuH.. (2008). Nerve growth factor helps protect retina in experimental retinal detachment. Ophthalmologica 222, 58–61. doi: 10.1159/000109281, PMID: 18097183

[ref31] TeleginaD. V.KolosovaN. G.KozhevnikovaO. S. (2019). Immunohistochemical localization of NGF, BDNF, and their receptors in a normal and AMD-like rat retina. BMC Med. Genet. 12:48. doi: 10.1186/s12920-019-0493-8, PMID: 30871541 PMC6417162

[ref32] UekiY.RehT. A. (2013). EGF stimulates muller glial proliferation via a BMP-dependent mechanism. Glia 61, 778–789. doi: 10.1002/glia.22472, PMID: 23362023 PMC4007577

[ref33] WakabayashiT.FujiwaraM.SakaguchiH.KusakaS.OshimaY. (2010). Foveal microstructure and visual acuity in surgically closed macular holes: spectral-domain optical coherence tomographic analysis. Ophthalmology 117, 1815–1824. doi: 10.1016/j.ophtha.2010.01.017, PMID: 20472291

[ref34] WanJ.RamachandranR.GoldmanD. (2012). HB-EGF is necessary and sufficient for Müller glia dedifferentiation and retina regeneration. Dev. Cell 22, 334–347. doi: 10.1016/j.devcel.2011.11.020, PMID: 22340497 PMC3285435

[ref35] WanJ.ZhaoX. F.VojtekA.GoldmanD. (2014). Retinal injury, growth factors, and cytokines converge on β-catenin and pStat3 signaling to stimulate retina regeneration. Cell Rep. 9, 285–297. doi: 10.1016/j.celrep.2014.08.048, PMID: 25263555 PMC4194164

[ref36] WangS.XuL.JonasJ. B. (2006). Prevalence of full-thickness macular holes in urban and rural adult Chinese: the Beijing eye study. Am. J. Ophthalmol. 141, 589–591. doi: 10.1016/j.ajo.2005.10.021, PMID: 16490523

[ref37] WuA. L.LiuY. T.ChouH. D.ChuangL. H.ChenK. J.ChenY. P.. (2021). Role of growth factors and internal limiting membrane constituents in muller cell migration. Exp. Eye Res. 202:108352. doi: 10.1016/j.exer.2020.108352, PMID: 33166502

[ref38] ZalisM. C.JohanssonS.Englund-JohanssonU. (2017). Immunocytochemical profiling of cultured mouse primary retinal cells. J. Histochem. Cytochem. 65, 223–239. doi: 10.1369/0022155416689675, PMID: 28151698 PMC5407564

[ref39] ZhangL.LiX.LinX.WuM. (2019a). Nerve growth factor promotes the proliferation of muller cells co-cultured with internal limiting membrane by regulating cell cycle via Trk-a/PI3K/Akt pathway. BMC Ophthalmol. 19:130. doi: 10.1186/s12886-019-1142-x, PMID: 31208396 PMC6580575

[ref40] ZhangL.LiX.ShenY.LinX.WuM. (2019b). Transdifferentiation effects and related mechanisms of nerve growth factor and internal limiting membrane on muller cells. Exp. Eye Res. 180, 146–154. doi: 10.1016/j.exer.2018.12.005, PMID: 30578789

